This article has been retracted.

# Study on the Mechanism of Treating Femoral Head Necrosis with Drynariae Rhizoma Based on Network Pharmacology

**DOI:** 10.1155/2022/3631722

**Published:** 2022-06-06

**Authors:** Luqing He, Chenyu Ma, Shuiqi Cai, Ruolin Hou, Hongfeng Xu, Jianqiang Liu, Xin Liu, Qun Huang

**Affiliations:** ^1^Central Laboratory of Traditional Chinese Medicine Orthopaedics, Third People's Hospital of Cixi, China; ^2^Department of Critical Care Medicine, Third People's Hospital of Cixi, China; ^3^Department of Orthopedics and Traumatology of Traditional Chinese Medicine, Third People's Hospital of Cixi, China; ^4^Department of Pharmacy, Third People's Hospital of Cixi, China; ^5^Department of General Surgery, Third People's Hospital of Cixi, China; ^6^Department of Rehabilitation, Third People's Hospital of Cixi, China

## Abstract

Through the network pharmacology thought, the action target of the active ingredients of Drynariae Rhizoma was predicted, and the mapping was combined with the related targets of ONFH, and the key nodes of interaction were identified for enrichment analysis, so as to comprehensively explore the pharmacological mechanism of Drynariae Rhizoma against ONFH. The main active ingredients of Drynariae Rhizoma were screened based on pharmacokinetic characteristics in pharmacokinetic database and analysis platform of TCM system (TCMSP). We used the organic small molecule bioactivity database (PubChem) and Swiss target prediction database to predict related targets based on 2D or 3D structural similarity and then mined the known ONFH therapeutic targets through the Human Mendelian Genetic Database (OMIM) and Pubmed texts. Combined with the predicted targets, String database was imported to construct the OP target interaction network diagram of bone fracture therapy. CytoNCA software was used to topology the key nodes of interaction according to relevant node parameters, and String was imported again to construct the protein interaction network diagram. Finally, biological functions and metabolic pathways of key nodes were analyzed through DAVID database. It was revealed that Drynariae Rhizoma may regulate stem cells, osteoblasts, osteoclasts, and immune cells through multiple pathways, including proliferation, differentiation, immunity, and oxidative stress. *Conclusion*: Pharmacological studies based on network indicate that Drynariae Rhizoma may participate in the regulation of several major signaling pathways through direct or indirect action targets and affect the proliferation and differentiation of multiple types of cells, thus playing an anti-ONFH role, which provides a scientific basis for explaining the material basis and mechanism of its anti- ONFH.

## 1. Introduction

Osteonecrosis necrosis of the femoral head (ONFH), one of the most common orthopedic diseases, is a disease caused by blood circulation disorder of the femoral head. Therefore, it is also called femoral head ischemic necrosis. The pathological changes are mainly bone cell blood loss, degeneration, and necrosis. The main changes in imaging are trabecular fracture and femoral head collapse. Long-term pathological changes will cause degenerative changes of articular cartilage and lead to joint inflammation, especially inflammatory lesions of the hip joint, which will cause pain and stiffness of the hip joint, limited activity, claudication, and other symptoms and eventually lead to the loss of hip joint function [1, 2]. The high incidence of femur head necrosis ranged from 30 to 65 years old, and male was higher than female. The high disability rate of femoral head necrosis will bring heavy burden to the patient's family and society.

Drynariae Rhizoma [3] is the dry rhizome of *Drynaria fortunei*, an orthopedic plant of Polypodiaceae. It has a warm and bitter taste, enters the liver and kidney meridian, and has the function of tonifying kidney and strengthening bone, healing pain, and relieving pain. It is used for the diseases of falling, falling, falling, broken bones, kidney deficiency and waist pain, weak bones and muscles, etc. Modern pharmacological studies have confirmed that Drynariae Rhizoma can promote the proliferation and differentiation of osteoblasts, promote bone regeneration of femoral head, inhibit the activity of osteoclasts, promote bone absorption of calcium, regulate blood calcium and phosphorus levels, and improve the internal environment of femoral head [4, 5]. At the same time, it was reported that total flavonoids of Rhizoma Drynariae have strong anti-osteonecrosis effect on knee hormone-induced femoral head. Experiments have shown that total flavonoids of Rhizoma Drynariae reduce cartilage lesions and significantly reduce Mankin cartilage integral [6], but its pharmacodynamic substance basis and mechanism of action are not clear.

In 2007, Hopkins proposed the term “network Pharmacology” [7]. Based on the “disease gene target drug” action network, it systematically observes the intervention and influence of drugs on the disease network and provides an effective strategy for the study of traditional Chinese medicine and compound prescription. Its integrity and systematicness are the same as the holistic view and dialectical treatment of “unity of heaven and man” in traditional Chinese medicine and the principle of multicomponent, multisystem, and multitarget synergy of traditional Chinese medicine and compound prescription. Therefore, this paper will use the method of network pharmacology to explore the anti ONFH mechanism of Drynariae Rhizoma, so as to provide a reference basis for the in-depth study of the anti ONFH effect of Drynariae Rhizoma.

## 2. Methods

### 2.1. Collection of Chemical Constituents from Drynariae Rhizoma

The traditional Chinese Medicine System Pharmacology (tcmsp) and the analysis platform (http://lsp.nwu.edu.cn/tcmsp.php) were used to search the chemical components of Drynariae Rhizoma. The molecular structure was obtained from PubChem database (http://pubchem.Ncbi.Nlm.nih.gov//) and saved in smiles format.

### 2.2. Active Ingredient Screening

ADME refers to the process of absorption, distribution, metabolism, and excretion of exogenous compounds by the organism. Evaluation of ADME is a key step in drug discovery and development. The vast majority of Chinese herbal medicines contain up to 50 or even thousands of compounds, but only a few compounds show ADME characteristics with potential biological effects [8]. Therefore, it is urgent to evaluate the effects and risks of Chinese herbal medicines on human body. Oral bioavailability (OB), one of the most common pharmacokinetic parameters in drug screening, refers to the rate and degree at which the effective ingredients of a drug are absorbed by the body and play a role [9]. Drug-likeness (DL) means the similarity of the functional group and physical properties between the compound and the known drug [10]; the greater the DL is, the more similar the compound is to the known drug, and DL ≥0.18 is usually the screening criterion [11]. OB ≥30% and DL ≥0.18 were selected as screening conditions in this study.

### 2.3. Prediction of the Target of Drynariae Rhizoma

Swiss database (http://www. Swiss target prediction.ch/) can accurately predict the target of the active ingredient based on the similarity between the 2D and 3D structure of the molecule and the known ligand [12]. SMILES were input into Swiss in turn, and “human” was taken as the research species to obtain the action target of bone fragment.

### 2.4. Disease Target Acquisition

Osteoporosis was searched through the Disgenet database (http://www.Disgenet.org/) to obtain the related genes and target proteins of ONFH. Potential targets for ONFH treatment were obtained by mapping with the above targets.

### 2.5. Construction of “ Drynariae Rhizoma – Active Compounds – Potential Action Targets” Network

The above active compounds and potential targets were introduced into Cytoscape, and the network of “ Drynariae Rhizoma – active compounds – potential targets” was drawn. The node represents Drynariae Rhizoma, active compounds, and potential targets, and the edge shows the relationship between the three. Conduct topology analysis on the network through the “network analyzer” plug-in, and set the network style according to the node connectivity (degree) and betweenness centrality. The node size reflects the degree size, and the thickness of the edge reflects the betweenness centrality.

### 2.6. Construction of Protein-Protein Interaction Network

The String database (Search tool for the Retrieval of Intervening genes, http://string-db. org/) has collected a large number of protein interactions obtained through experimental detection and bioinformatics methods, involving a total of 9 643 763 proteins and 1 380 838 440 interactions [13]. The potential target of ONFH treatment by bone fragment was imported into String, and the species was selected as “human” to obtain protein interaction information, and the note1, note2, and Combine score information were imported into Cytoscape to draw protein interaction.

### 2.7. Biological Function and Pathway Enrichment Analysis of the Target

The DAVID database (Database for Annotation, Visualization and Integrated Discovery, https://David.ncifcrf.gov/) is a high-throughput biological information annotation database, which can provide systematic and comprehensive biological function annotation information for large-scale genes or proteins, so as to mine their biological significance [14]. The potential targets were imported into David database, and the species were defined as “human” for GO gene ontology-biological process and KEGG Pathway enrichment analysis. The biological processes with *P* < 0.01 and signaling pathways with *P* < 0.05 were screened and mapped with Origin 2018.

## 3. Results

### 3.1. The Active Constituents and Molecular Structure of Drynariae Rhizoma

A total of 71 compounds were collected, and 18 active components were screened according to OB ≥30% and DL ≥ 0. 18 (Table 1).

### 3.2. Potential Targets of Drynariae Rhizoma against ONFH

A total of 141 predicted targets were obtained by combining the predicted targets obtained from Swiss database. A total of 464 ONFH disease targets were obtained by searching Disgenet database. A total of 24 potential targets against ONFH were obtained by phase mapping.

### 3.3. The Network of “ Drynariae Rhizoma – Active Compounds – Potential Targets”

The active compounds and potential targets were introduced into Cytoscape to obtain a network of “ Drynariae Rhizoma – active compounds – potential targets,” as shown in Figure 1. And it turns out that the ingredients stigmasterol, beta-sitosterol, eriodyctiol (flavanone), kaempferol, naringenin eriodictyol, cycloartenone, and eriodictyol can bind to more than 5 targets and are the main components of bone fragment anti-ONFH. The target CYP19A1 was linked with the components 8 times, which was of great significance for anti-ONFH of bone fragment. CYP1B1 was 4 times, and MMP1, CA2, CYP17A1, ESR1, MMP13, LDLR, CYP1A1, and MMP2 were all 3 times, which had great significance for the anti-ONFH of bone fragment.

### 3.4. Predicting the Target of Active Components of Drynariae Rhizoma

The target prediction of 16 chemical components of Drynariae Rhizoma was carried out through Swiss target prediction. The screening possibility was high, and a total of 118 targets were obtained after weight removal. KEGG enriched 32 signal pathways and constructed compound target interaction network by Cytoscape, as shown in Figure 2.

### 3.5. Screening and Construction of Key Nodes of Drynaria Drynariae Acting on ONFH and PPI Network Diagram

The target target (T-T) interaction network is constructed through string, with 393 nodes and 5201 relationships. After screening according to DC, BC, CC, EC, NC, lac, and other topologies by cytonca, 97 key nodes and 2332 relationships are obtained, and string is imported again to construct PPI network (see Figure 3).

### 3.6. Enrichment Analysis of Key Nodes of Drynariae Rhizoma Acting on ONFH

After go enrichment analysis of key nodes in David database (*P* < 0.05), a total of 320 enrichment results were obtained. It includes 255 items of biological process (BP), 39 items of molecular function (MF), and 26 items of cellular component (CC). The enrichment results of GO in the top five are shown in Figure 4. KEGG enriched 109 pathways. The top ranked major related signaling pathways of ONFH are PI3K/Akt signalling pathway, Wnt signaling pathway, estrogen signaling pathway, mitogen-activated protein kinase (MAPK) signaling pathway, osteoclast differentiation, signaling pathways that can regulate pluripotency in stem cells, FOXO signaling pathway, tumor necrosis factor (TNF) signaling pathway, thyroid hormone signaling pathway, Rap1 signaling pathway, and other pathways.

## 4. Discussion

At present, there are many clinical treatment methods for ONFH, including oral and external use of traditional Chinese medicine and Western medicine, protective weight-bearing, hip preserving surgery, interventional therapy, hyperbaric oxygen, extracorporeal shock wave, and artificial joint replacement. Patients in the early and middle stage mostly take nonsurgical treatment, and patients in the late stage mostly choose surgical treatment. Traditional medicine believes that the kidney is the foundation of congenital, the kidney governs the bone, the bone generates marrow, and the kidney essence is the foundation of one's life, which determines human growth, development, and reproduction. The clinical syndrome of ONFH mostly belongs to deficiency of kidney essence, so the treatment is mainly to tonify the kidney. Drynariae Rhizoma is the dry rhizome of Polypodiaceae plant quercetin. It is a commonly used traditional Chinese medicine in orthopedics and traumatology for the treatment of ONFH [15, 16]. The regulatory system in the body is usually not the core of a single data signaling pathway, but an intricate network of controls. Different data signaling pathways and targets all have certain degree of signal transduction, so the relevant components of drugs not only mainly combine with component targets at the same time, but also directly or indirectly bind with other targets.

In this study, we found that 50 active chemicals were common targets among the 118 predicted and analyzed targets, reflecting the synergistic effect of multiple components of Drynariae Rhizoma, which also played a key role in the pathogenesis of ONFH. Aggregation analysis of predictive analysis targets showed that after removing common pathways, the top pathways included cell cycle pathway, estrogen pathway, calcium pathway, and inflammatory data signaling pathway, which were closely related to the development trend of ONFH. Basically, this study suggests that the active ingredients of Drynariae Rhizoma have the potential to exert their comprehensive anti-ONFH effects in a variety of ways.

From the key topology nodes, aromatase (CYP19A1), estrogen receptor 1 (ESR1), cytochrome P450, family 1, subfamily A, polypeptide 1 (CYP1A1), matrix metalloproteinase 2 (MMP-2), androgen protein kinase (AR), chemokine receptor 2 (CCR2), and matrix metalloproteinase 3 (MMP-3) are both ONFH targets and predictive analysis targets of the components related to bone fragment. This connection point may be the target of ONFH simultaneous action of bone splice. Eighty-seven index values were independently associated with Drynariae Rhizoma or ONFH, and three of them were neither predictive analysis index values nor ONFH related index values. ONFH can be applied to ONFH using simultaneous or indirect index values. The results of GO aggregation analysis showed that the effect of Drynariae Rhizoma on ONFH might be related to the whole process of BP, such as immunity, inflammation, capillary transformation, and cell necrosis. MF level indicated that cell growth factor, adenosine triphosphate (ATP), transcription factors, and other molecules fully play the role of anti-ONFH. CC level indicates that the system almost covers all the steps of data signaling pathway from production to recovery, such as extracellular, cytoplasmic, nuclear, cytoplasmic, transcription factor complex, Golgi body, and exosome.

KEGG summarized and analyzed the key nodes and further revealed that the osteoclast is based on a variety of methods, from proliferation, differentiation, and immunity, and from multiple levels, such as the regulation of oxidative stress on stem cells, osteoblasts and osteoclasts, and cellular immunity. The classical Wnt data signaling pathway plays a bidirectional role in the differentiation of osteoblasts and osteoclasts. Inflammatory factors play a major role in the ONFH system [15, 16]. The enhancement of inflammatory factors caused by various factors can increase the number of osteoclasts, inhibit osteogenesis, and promote bone cell necrosis. FoxO pathway plays a major role in the antioxidative stress state, and FoxO3 and FoxO4 genes can reduce the total number of osteoblasts in bone and increase the level of inflammatory factors [17]. Meanwhile, FoxO is a transcription factor closely related to Wnt/*β*-catenin, and the signal of Wnt antagonism increases with time. Estrogen data signaling pathway plays a major role in the production of ONFH after amenorrhea, and the reduction of estrogen data signaling pathway can lead to the promotion of osteoclast and the increase of osteoclast activity on the one hand [18]. On the other hand, it promotes the metabolism of inflammatory factors such as interleukin and TNF family, leading to osteoclast differentiation and stimulating osteoclast activity [19]. Rap1 is particularly important for bone resorption, and selective inhibition of its expression in perfecting osteoclasts can slow down physiological bone loss [20]. Studies have shown that Rap1 acts as a molecular power switch based on the conversion of two fusion conformation of guanosine diphosphate (GDP) and calcium triphosphate active guanosine (GTP), involving PI3K/Akt downstream. P38 MAPK and other ways can impair bone metabolism. Activation of PI3K/Akt data signaling pathway can stimulate osteoblast proliferation and differentiation and inhibit cell necrosis [21]. Studies have found that active MAPK plays an important role in increasing osteoblast production, reducing osteoclast differentiation, and improving ONFH level [22–24]. The thyroxine pathway can affect the progression of ONFH by affecting the proliferation and differentiation of osteoblasts and osteoclasts [25, 26]. These results indicate that Drynariae Rhizoma can play a role in ONFH through the targets and levels of the signal pathway network of the mainstream as well as the indirect target receptors [27–30]. It further indicated the advantages of Drynariae Rhizoma in the treatment of ONFH, which has great potential for drug research and development. However, its main regulatory mechanism still needs further experimental verification.

Due to the complexity of the effective components of Chinese medicinal materials and the limitations of experimental research ideas, there is still a lack of investigation reports on the chemical targets and the effectiveness of ONFH alone. This analysis, using network pharmacology, is the first to decipher the potential active ingredients of Drynariae Rhizoma, which can be based on the multitarget, multimode, multisystem important molecular structure in the efficacy of ONFH. As there are totally 16 active ingredients and 55 key targets of Drynariae Rhizoma in treating ONFH (Table 2), no database could perform the high throughout molecular docking analysis for the above targeting. This is the limitation of this study.

Network pharmacology is widely used in life science research in the fields of drugs, target identification, lead compound discovery, mechanism of action analysis, clinical research, efficacy, and safety factors. Based on the prediction and analysis of network pharmacology, we can analyze the relevant chemical substances, potential therapeutic targets, and key signaling pathways for the treatment of ONFH or select reasonable components for molecular docking simulation and then quantitatively analyze the fingerprints to establish a scientific, rational, and easy-to-use basis for multi-indicator evaluation, providing a basis for future relevant scientific research.

## Figures and Tables

**Figure 1:** The network of “ Drynariae Rhizoma – active compounds – potential targets”.

**Figure 2:** Network of 16 active compounds of Rhizoma Drynariae and 118 putative targets.

**Figure 3:** Network of 97 key nodes based on their direct interactions.

**Figure 4:** GO and KEGG enrichment analysis of key targets.

**Table 1:** Potential active compounds in Drynariae Rhizoma with OB and DL parameters.

mol ID	Compound name	Structural information	OB%	DL
5280445	Luteolin	2-(3,4-dihydroxyphenyl)-5,7-dihydroxychromen-4-one	36.16	0.25
222284	Beta-sitosterol	24-ethylcholest-5-en-3 beta-ol	36.91	0.75
101729	Cyclolaudenol	15-(5,6-dimethylhept-6-en-2-yl)-7,7,12,16-tetramethyl-6-pentacyclo	39.05	0.79
91692436	22-Stigmasten-3-one	17-[(E,2R,5R)-5-ethyl-6-methylhept-3-en-2-yl]-10,13-dimethyl-tetradecahydrocyclopenta	39.25	0.76
12305360	Cycloartenone	7,7,12,16-tetramethyl-15-[(2R)-6-methylhept-5-en-2-yl]pentacyclo	40.57	0.79
14309735	Xanthogalenol	[2,6-dihydroxy-4-methoxy-3-(3-methylbut-2-enyl)phenyl]-3-(4-hydroxyphenyl)prop	41.08	0.32
373261	Eriodyctiol (flavanone)	(2R)-2-(3,4-dihydroxyphenyl)-5,7-dihydroxy-2,3-dihydrochromen-4-one	41.35	0.24
6427354	Cyclolaudenol acetate	15-(5,6-dimethylhept-6-en-2-yl)-7,7,12,16-tetramethyl-6-pentacyclo[9,8.012,16] acetate	41.66	0.79
5280863	Kaempferol	3,5,7-trihydroxy-2-(4-hydroxyphenyl)chromen-4-one	41.88	0.24
667495	(2R)-5,7-dihydroxy-2-(4-hydroxyphenyl)chroman-4-one	(2R)-5,7-dihydroxy-2-(4-hydroxyphenyl)chroman-4-one	42.36	0.21
5280794	Stigmasterol	10,13-dimethyl-14,15,16,17-dodecahydro-1H-cyclopenta[a]phenanthren-3-ol	43.83	0.76
5281220	Aureusidin	[(3,4-dihydroxyphenyl)methylidene]-4,6-dihydroxy-1-benzofuran-3-one	53.42	0.24
9064	(+)-catechin	(2R,3S)-2-(3,4-dihydroxyphenyl)-3,4-dihydro-2H-chromene-3,5,7-triol	54.83	0.24
932	Naringenin	5,7-dihydroxy-2-(4-hydroxyphenyl)-2,3-dihydrochromen-4-one	59.29	0.21
54711004	Digallate	4-(5-carboxy-2,3-dihydroxyphenoxy)carbonyl-2,6-dihydroxyphenolate	61.85	0.26
44257070	Davallioside A_qt	5,7-dihydroxy-3-[(2R,5S,6R)-3,4,5-trihydroxy-6-(hydroxymethyl)oxan-2-yl]oxy-3,4-dihydro-2H-chromen-8-yl]pyrrolidin-2-one	62.65	0.51
10411827	Marioside_qt	3,4,5-trihydroxy-6-methyloxan-2-yl]oxymethyl]oxane-2,3,4,5-tetrol	70.79	0.19
440735	Eriodictyol	(2S)-2-(3,4-dihydroxyphenyl)-5,7-dihydroxy-2,3-dihydrochromen-4-one	71.79	0.24

**Table 2:** Active ingredients and key targets of Drynariae Rhizoma in treating ONFH.

No.	Active ingredients	Key targets
1	Luteolin	MMP1, MMP2, and MMP13
2	Beta-sitosterol	AR, CYP19A1, CYP17A1, LDLR, ESR1, and ESR2
3	Cyclolaudenol	LDLR, HSD11B1, and UGT2B17
4	22-Stigmasten-3-one	TRPV1, TRPV4, and CYP19A1
5	Cycloartenone	CYP19A1, TRPV1, TRPV4, CYP17A1, and NR3C1
6	Xanthogalenol	CYP19A1 and NOS3
7	Eriodyctiol (flavanone)	CYP1B1, CYP1A1, CYP19A1, MMP1, and MMP13
8	Kaempferol	ABCB1, HSD17B1, ALOX15, ALOX12, and CYP1B1
9	Stigmasterol	AR, CYP19A1, LDLR, CYP17A1, ESR1, and ESR2
10	Aureusidin	ERBB2
11	(+)-catechin	CA2
12	Naringenin	CYP19A1, HSD17B1, CYP1B1, CYP1A1, and ESR1
13	Digallate	CA2
14	Davallioside A_qt	MMP2 and CA2
15	Marioside_qt	STAT1 and MMP2
16	Eriodictyol	CYP1B1, CYP1A1, CYP19A1, MMP1 and MMP13

## Data Availability

The data used to support this study are available from the corresponding author upon request.
